The article "Network-Based Elaboration of the Efficacy of the Dachangshu (BL25) and Tianshu (ST25) Points in the Treatment of Functional Constipation in Children through Inflammation, Adipocytokine, or Leptin Pathways" was retracted in 2023. Reasons: signs of a paper mill; suspected computer-generated content; unreliable results or conclusions; concerns about the data.

# Network-Based Elaboration of the Efficacy of the Dachangshu (BL25) and Tianshu (ST25) Points in the Treatment of Functional Constipation in Children through Inflammation, Adipocytokine, or Leptin Pathways

**DOI:** 10.1155/2022/5315927

**Published:** 2022-12-06

**Authors:** Yan Xu, Hanying Xu, Xinna Wang, Hongjuan Wen, Huifang Guan, Fa Gao, Hang Xu, Wei Jing, Jing Li, Yan Mei, Weibin Li, Qixiong Chen, Fang Liu, Hongtao Cui

**Affiliations:** ^1^School of Pediatrics, Henan University of Chinese Medicine, Zhengzhou, Henan 450000, China; ^2^The First Affiliated Hospital of Henan University of Chinese Medicine, Zhengzhou, Henan 450000, China; ^3^Changchun University of Chinese Medicine, Changchun, Jilin 130117, China; ^4^Chongqing Hospital Of Traditional Chinese Medicine, Chongqing 400021, China

## Abstract

Constipation commonly occurs during childhood, and more than 95% of cases are classified as functional constipation. If not effectively treated, 20% of patients with childhood constipation can continue to exhibit symptoms into adulthood, which seriously affects their mental health and quality of life. The main feature of acupuncture or acupoint stimulation, a special branch of traditional Chinese medicine, is the selection of different acupoints for different diseases, and many worthy guidelines have been established for matching acupoints. The back-shu and front-mu point combination adheres to an important acupoint compatibility law that has been used since its proposal 2,500 years ago but has not yet been verified by the modern evidence-based experiments. This study focused on the back-shu and front-mu point combination using the Dachangshu (BL25) and Tianshu (ST25) points as examples to explore possible research methods for network acupoint-based stimulation based on existing evidence and to elucidate the mechanisms induced by BL25 and ST25 in the treatment of functional constipation in children (FCC). The study found that BL25 and ST25 have 20 common targets, namely, AQP8, DRD2, VIP, TAC1, IL6R, TNF, FOS, KIT, CHAT, HTR3A, GAS8, SOD3, TRPV1, MPO, CALCA, IL1B, P2RX7, NPY2R, IL10RA, and TPH1, and these targets may provide a strategy for the combined usage of BL25 and ST25. In addition, BL25 and ST25 can affect FCC treatment through inflammation-relatedTh17-cell differentiation, the NF-kappa B signaling pathway, and the Toll-like receptor signaling pathway. Adipocytokines or leptin may also comprise the mechanism through which BL25 and ST25 regulate FCC. In addition, BL25 and ST25 regulate FCC through 13 core targets, namely, NFKBIA, RELA, TNF, IKBKB, IRAK1, TLR4, MYD88, TNFRSF1A, IL1R1, TLR2, IL1B, TRAF6, and TNFRSF1B. In short, this study provides new ideas and methods for studying the mechanism of acupuncture points.

The article "Network-Based Elaboration of the Efficacy of the Dachangshu (BL25) and Tianshu (ST25) Points in the Treatment of Functional Constipation in Children through Inflammation, Adipocytokine, or Leptin Pathways" was retracted in 2023. Reasons: signs of a paper mill; suspected computer-generated content; unreliable results or conclusions; concerns about the data.

## 1. Background

Constipation commonly occurs during childhood, with an incidence ranging from 3% to 30%, and more than 95% of all cases are classified as functional constipation [1]. The median age of constipation onset in children is 2.3 years, and the ages at the 25th and 75th percentiles are 0.8 and 4.8 years, respectively [2]. If not effectively treated, 20% of patients with childhood constipation continue to exhibit symptoms into adulthood, which seriously affects their mental health and quality of life [3]. Therefore, early intervention for functional constipation in children (FCC) is necessary to reduce the impacts on mental health and quality of life in adulthood.

The traditional Chinese medicine (TCM) theory has gradually developed over a long period based on medical practices guided by ancient simple Chinese material principles and dialectics of nature and includes complex theoretical systems and treatment methods. Acupuncture or acupoint stimulation is a special branch of TCM. The selection of different points for different diseases is the main feature of acupuncture or acupoint stimulation, and many important laws have been established for matching acupoints. A typical method is the back-shu and front-mu point combination, which has been considered the classic acupoint combination applied in the clinic since its proposal in the “Classic of Questioning” 2500 years ago and is still used today. Simply, the back-shu and front-mu point combination is based on the yin and yang theory in Chinese medicine. The abdomen (which belongs to yin according to the TCM theory) and the back (which belongs to yang according to the TCM theory) are selected as acupoint stimulation targets to balance yin and yang and thereby regulate visceral functions. Some studies have investigated the regulatory mechanisms of the back-shu and front-mu points, including the Feishu point (back-shu point) and the Zhongfu point (front-mu), which can reduce inflammatory exudation and inflammatory cell infiltration in the lung tissues of asthmatic mice [4]. The Weishu point (back-shu point) and Zhongwan point (front-mu) can regulate gastric motility and are closely related to the thalamus, limbic system, and some brain areas of the default network [5]. The Dachangshu point (BL25, back-shu point) and Tianshu point (ST25, front-mu point) regulate the expression of c-kit and TRPV1 to improve diarrhea in rats with an irritable bowel syndrome [6]. However, most studies are limited to the investigation of a single mechanistic change after acupoint stimulation and cannot explain the complex multimechanistic and multifunctional changes that subsequently occur in the human body. To more specifically explain the relatively complex mechanistic changes that occur after acupuncture point stimulation, we assessed the combination of BL25 (back-shu point) and ST25 (front-mu) in the treatment of FCC and explored the complex mechanism induced by acupoint stimulation based on existing evidence.

The article "Network-Based Elaboration of the Efficacy of the Dachangshu (BL25) and Tianshu (ST25) Points in the Treatment of Functional Constipation in Children through Inflammation, Adipocytokine, or Leptin Pathways" was retracted in 2023. Reasons: signs of a paper mill; suspected computer-generated content; unreliable results or conclusions; concerns about the data.

BL25 was selected as the research object because it belongs to the bladder meridian of foot-taiyang, which is also the dorsal point of the large intestine. BL25 is located at the same level as the inferior border of the spinous process of the fourth lumbar vertebra (L4), 1.5 B-cun lateral to the posterior median line. According to the TCM theory, targeting BL25 can cure abdominal pain, bloating, diarrhea, and constipation, among other ailments. Previous studies have provided ample information about BL25, and the evidence shows that targeting this point can enhance jejunal movement in rats with constipation and diarrhea [7], that moxibustion at BL25 can reduce visceral hyperalgesia [8] and that electroacupuncture at BL25 can be used to treat inflammatory bowel disease (IBD) in mice [9]. ST25 belongs to the stomach meridian of foot-yangming, the front-mu acupoint of the large intestine. ST25 is located on the upper abdomen, 2 B-cun lateral to the center of the umbilicus. ST25 can be used to treat many of the same ailments as BL25, including abdominal pain, bloating, diarrhea, and constipation. Previous studies on ST25 have revealed that this acupoint can be targeted to treat functional constipation [10], that acupuncture at ST25 is safe and effective for the treatment of functional constipation [11] and that the moxibustion of ST25 can exert its effect on TNBS-induced colitis rats by triggering the degranulation of local mast cells [12], among other effects. Some clinical evidence, including the results from Zhu Qi's clinical research on stimulating BL25 and other back-shu points to treat senile constipation through warm needling moxibustion, demonstrates that the total effective rate of stimulating back-shu points to treat senile constipation is higher than that of ordinary acupuncture [13]. Guifang and Yuejuan used iontophoresis to stimulate ST25 and BL25 in a clinical study of stroke patients and found that the improvement rate in the symptom score obtained through stimulation at ST25 combined with BL25 was higher than that obtained with conventional treatment [14]. Hui et al.'s clinical observation of 40 patients with functional constipation treated with acupuncture at BL25 and ST25 also found that the number of stools from patients treated with BL25 and ST25 was significantly increased [15]. In addition, some studies have investigated FCC. For example, Niansong et al. used pediatric massage combined with acupoint stimulation (including ST25) to treat 75 cases of FCC and found that the symptom score decreased after treatment, which showed that pediatric massage combined with acupoint stimulation can significantly improve the clinical symptoms of FCC [16]. Although the abovementioned studies showed that BL25 and ST25 can be widely used in the treatment of intestinal diseases, no comprehensive or systematic evidence-based analyses of these two acupoints in the treatment of FCC have been performed.

The article "Network-Based Elaboration of the Efficacy of the Dachangshu (BL25) and Tianshu (ST25) Points in the Treatment of Functional Constipation in Children through Inflammation, Adipocytokine, or Leptin Pathways" was retracted in 2023. Reasons: signs of a paper mill; suspected computer-generated content; unreliable results or conclusions; concerns about the data.

In brief, this study aimed to assess the back-shu and front-mu point combination using BL25 and ST25 as examples to explore network acupoint research methods based on existing evidence and to elucidate the mechanisms induced by stimulation at BL25 and ST25 in the treatment of FCC. The results of this study should provide new ideas and methods for acupuncture research. The research route is shown in Figure 1.

## 2. Materials and Methods

### 2.1. Retrieval of Information on BL25 and ST25 Targets

We manually searched the CNKI, Wanfang, VIP, PubMed, and Web of Science databases to collect information on targets of BL25 and ST25, and the search time was from the time of database creation to July 1, 2021. Using a search method involving subject headings and free words and taking a PubMed search based on BL25 as an example, the search formula was (((((((((((((((((((((((((((Acupuncture Points [MeSH Terms])) OR (Electroacupuncture [MeSH Terms])) OR (Moxibustion [MeSH Terms])) OR (Acupuncture Therapy [MeSH Terms])) OR (Acupuncture Point)) OR (Point, Acupuncture)) OR (Points, Acupuncture)) OR (Acupoints)) OR (Acupoint)) OR (Acupuncture Treatment)) OR (Acupuncture Treatments)) OR (Treatment, Acupuncture)) OR (Therapy, Acupuncture)) OR (Pharmacoacupuncture Treatment)) OR (Treatment, Pharmacoacupuncture)) OR (Pharmacoacupuncture Therapy)) OR (Therapy, Pharmacoacupuncture)) OR (Acupotomy)) OR (Acupotomies)) AND (((BL25) OR (B25)) OR (Dachangshu)). Reexamination, debugging, double-checking, and omission repair were performed by special personnel.

### 2.2. Correction of BL25 and ST25 Target Names

The two acupoint targets were entered separately into the UniProt database (https://www.UniProt.org/) for correction and conversion into gene names. UniProt is a nonredundant protein sequence database with the most complete sequence data and the richest annotation information in the world. Since its establishment at the beginning of this century, this database has provided valuable resources for the field of life sciences. More than 500,000 sequences in the Swiss-Prot sublibrary were manually reviewed and annotated, and all corrected data in this study were obtained from the Swiss-Prot sublibrary. The target information for the two acupoints was then uploaded to the website (https://www.tcmmodel.com).

The article "Network-Based Elaboration of the Efficacy of the Dachangshu (BL25) and Tianshu (ST25) Points in the Treatment of Functional Constipation in Children through Inflammation, Adipocytokine, or Leptin Pathways" was retracted in 2023. Reasons: signs of a paper mill; suspected computer-generated content; unreliable results or conclusions; concerns about the data.

### 2.3. FCC-Related Genes

The key phrase “functional constipation in children” was searched in the GeneCards database (https://www.genecards.org) to identify disease-related genes, and those related to both the acupoint targets and FCC were retained. Cytoscape 3.8.2 software was then used to prepare the figure.

### 2.4. KEGG and Local STRING Network Enrichment Analysis

The above-described genes were inputted into the String (https://string-db.org/) database, and their functional enrichment was assessed based on Kyoto Encyclopedia of Genes and Genomes (KEGG) and local STRING network clusters. A bioinformatics website (https://www.bioinformatics.com.cn) was then used to prepare the figure.

In the KEGG and local STRING network clusters, the strength was directly associated with the substantiality of the enrichment effect. The false discovery rate indicated the significance of the enrichment, and the *p* values for each category were subjected to multiple-testing correction using the Benjamini–Hochberg procedure.

The local STRING network cluster enrichment analysis included precomputed protein clusters derived from a hierarchical clustering of the full STRING network using an average linkage algorithm. The cluster names were derived automatically based on the consensus protein annotations from the GO, KEGG, Reactome, UniProt, Pfam, SMART, and InterPro databases. All clusters and their hierarchical tree are available for download in the download section of STRING (https://string-db.org/cgi/download.pl). In brief, local STRING network clusters were reenriched based on the STRING, GO, KEGG, Reactome, UniProt, Pfam, SMART, and InterPro databases, which may provide a more comprehensive description of the gene enrichment status. Therefore, we selected the local STRING network clusters for reenrichment.

We also used the following principles to select the enriched pathways: (1) pathways that have been proven to be directly or indirectly related to FCC; (2) pathways with the same or similar mechanisms present in both the enrichment methods; and (3) multiple pathways with the same or a similar meaning.

## 3. Results

### 3.1. BL25 and ST25 Target Information

After retrieval, removal of redundant data, and correction based on the UniProt database, a total of 56 BL25 targets and 122 ST25 targets were obtained, as shown in Figure 2. Twenty targets were shared between BL25 and ST25: AQP8, DRD2, VIP, TAC1, IL6R, TNF, FOS, KIT, CHAT, HTR3A, GAS8, SOD3, TRPV1, MPO, CALCA, IL1B, P2RX7, NPY2R, IL10RA, and TPH1.

The article "Network-Based Elaboration of the Efficacy of the Dachangshu (BL25) and Tianshu (ST25) Points in the Treatment of Functional Constipation in Children through Inflammation, Adipocytokine, or Leptin Pathways" was retracted in 2023. Reasons: signs of a paper mill; suspected computer-generated content; unreliable results or conclusions; concerns about the data.

### 3.2. FCC and Intersection Genes

After removing the redundancy among the BL25 and ST25 targets, an analysis of the FCC genes from the GeneCards database that intersected with the abovementioned targets revealed 115 targets that were related to the two acupoints and diseases. Detailed information is provided in Supplementary Material 1 and shown in Figure 3.

### 3.3. KEGG Enrichment Analysis

The abovementioned targets were entered into the STRING website, and the analysis function was used to obtain enrichment information for 141 KEGG pathways. Detailed information is provided in Supplementary Material 2. The strength values were sorted from high to low, and the first 20 pathways were selected for analysis (Figure 4). IBD, which mainly includes ulcerative colitis and Crohn's disease, was identified as the most important enriched item. IBD is a chronic nonspecific inflammatory disease involving the gastrointestinal tract that is recurring and difficult to treat [17]. In addition, the adipocytokine signaling pathway [18, 19], Th17-cell differentiation [20], NF-kappa B signaling pathway [21], and Toll-like receptor signaling pathway [22] may also be closely related to FCC.

### 3.4. Local STRING Network Cluster Enrichment Analysis

A total of 59 local STRING network cluster enrichment items were obtained, as shown in Supplementary Material 3. As shown in Figure 5, the I*κ*BA variant leads to EDA-ID; the I*κ*BA variant leads to EDA-ID and death-inducing signaling complex assembly; TAK1 activates NF-*κ*B by phosphorylation and activation of the IKK complex; and death-inducing signaling complex assemblies are closely related to the NF-*κ*B signaling pathway. The enrichment of local STRING network clusters also revealed that the NF-*κ*B signaling pathway is correlated with acupoints and FCC.

The enrichment analysis of the local STRING network clusters also showed several pathways that are related to inflammation, such as the interleukin-1 receptor complex and IRAK4 deficiency (TLR5); IRAK4 deficiency (TLR2/4) and interleukin-1 receptor complex; interleukin-1-mediated signaling pathway and TIR domain; MyD88 deficiency (TLR2/4); and MyD88-dependentToll-like receptor signaling pathway and interleukin-1 conserved site pathways. All of these pathways are related to IL-1 or MyD88; IL-1 is a well-known proinflammatory factor [23], and MyD88 is a key linker molecule in the Toll-like receptor signaling pathway. MyD88-dependentToll-like receptor signaling and the interleukin-1 conserved site pathway are closely related to the Toll-like receptor signaling pathway, which was found to be enriched by the KEGG analysis. Both IL-1 and MyD88 are closely related to rectal diseases [24], and MyD88 can mediate the proliferation, migration, and invasion of rectal cancer cells via the NF-*κ*B signaling pathway [25]. In addition, the orexin receptor family, prepro-orexin, leptin signaling, and erythropoietin activate phospholipase C gamma (PLCG) pathways and appear to have functions similar to that of the adipocytokine signaling pathway in the KEGG database, and these pathways function by regulating the neuropeptide levels.

The article "Network-Based Elaboration of the Efficacy of the Dachangshu (BL25) and Tianshu (ST25) Points in the Treatment of Functional Constipation in Children through Inflammation, Adipocytokine, or Leptin Pathways" was retracted in 2023. Reasons: signs of a paper mill; suspected computer-generated content; unreliable results or conclusions; concerns about the data.

In short, enrichment analyses of the KEGG and local STRING network clusters revealed two important points. First, the potential mechanisms through which the two acupoints regulate FCC appear to be related to inflammatory pathways, including the following: NF-*κ*B signaling, Toll-like receptor signaling, IKBA variant leads to death-inducing signaling complex assembly, TAK1 activation of NF-*κ*B by phosphorylation and activation of the IKK complex and death-inducing signaling complex assembly, interleukin-1 receptor complex, IRAK4 deficiency (TLR5), IRAK4 deficiency (TLR2/4), interleukin-1 receptor complex, interleukin-1-mediated signaling pathway, TIR domain, MyD88 deficiency (TLR2/4), MyD88-dependentToll-like receptor signaling pathway, and interleukin-1 conserved site pathways. Second, adipocytokines and leptin appear to be associated with the acupoint regulation of FCC, including through adipocytokine signaling, the orexin receptor family, prepro-orexin, and leptin signaling, and erythropoietin activates PLCG pathways.

Therefore, we subsequently aimed to analyze the abovementioned 13 signaling pathways to determine commonalities.

### 3.5. Signaling Pathway-Target Relationship Network

To identify the commonalities among the abovementioned 13 pathways, the pathway-target relationship network was constructed using Cytoscape. As shown in Figure 6, a total of 34 targets were included in the network, and the targets simultaneously participating in 4 or more pathways were considered the core targets. Thirteen targets were included, namely, NFKBIA, RELA, TNF, IKBKB, IRAK1, TLR4, MYD88, TNFRSF1A, IL1R1, TLR2, IL1B, TRAF6, and TNFRSF1B, and these were considered the core targets through which the BL25 and ST25 acupoints can treat FCC.

## 4. Discussion

### 4.1. The Combination of BL25 and ST25 May Enhance the Therapeutic Effect of a Single Acupoint

According to the TCM theory, the back-shu point refers to the acupoints at which the energies of the five internal organs and six FCs are inflicted upon the back. In subjects with visceral diseases, the corresponding back-shu points often have abnormal reactions, such as sensitivity and tenderness, and stimulation of these acupoints can be used to treat corresponding visceral diseases. BL25 corresponds to the passage of qi in the large intestine through the back, and stimulation of BL25 can regulate the pathological changes in the large intestine. Front-mu acupoints are those at which the vital energies of the viscera are infused into the chest and abdomen, and “mu” means gathering and confluence. Similar to the back-shu point, when the viscera are diseased, stimulation of the front-mu acupoint usually results in abnormal manifestations such as sensitivity and tenderness. ST25 is also the front-mu acupoint of the large intestine. In clinical treatment, the back-shu and front-mu points are often used in combination due to their similar effects. Despite being used for thousands of years, Chinese researchers have not provided evidence-based experimental results that sufficiently support the effectiveness of this combination therapy. This study aimed to analyze the existing evidence and revealed that BL25 and ST25 have 20 common targets, namely, AQP8, DRD2, VIP, TAC1, IL6R, TNF, FOS, KIT, CHAT, HTR3A, GAS8, SOD3, TRPV1, MPO, CALCA, IL1B, P2RX7, NPY2R, IL10RA, and TPH1. These targets may underlie how BL25 and ST25 can be used together to enhance the therapeutic effect. In addition, because the BL5 and ST25 combination is based on the specific embodiment of back-shu and front-mu points, other acupoints belonging to the back-shu and front-mu point combination may also have similar matching targets, and this possibility may represent a direction of future research on acupoint compatibility.

The article "Network-Based Elaboration of the Efficacy of the Dachangshu (BL25) and Tianshu (ST25) Points in the Treatment of Functional Constipation in Children through Inflammation, Adipocytokine, or Leptin Pathways" was retracted in 2023. Reasons: signs of a paper mill; suspected computer-generated content; unreliable results or conclusions; concerns about the data.

### 4.2. Mechanism through Which BL25 and ST25 Regulate FCC

FCC can be attributed to eating habits (too much milk or too little fiber), changes in the intestinal flora, and psychological and behavioral factors secondary to systemic diseases or drug use, among other factors [26]. Among these factors, the histological changes in the colonic mucosa caused by a milk protein allergy [27] and some diseases, such as colon cancer and IBD [28], are closely related to inflammation. Other diseases, including intestinal diseases, anorectal diseases, metabolic and endocrine diseases, neuropathological diseases, and other systemic diseases, are also causes of FCC [26]. In addition, FCC is more common in children with autism, attention-deficit hyperactivity disorder, anxiety, and depression than in healthy children [29–33].

In this study, KEGG and local STRING network cluster analyses revealed several interesting potential functions of BL25 and ST25.

#### 4.2.1. BL25 and ST25 Regulate FCC through Inflammation

Constipation is a common problem in childhood, affecting approximately 3% of children in the world, and up to 30% of children in some environments suffer from constipation. Constipation is defined as infrequent bowel movements (<2 times per week), reduced bowel frequency, occurrence of fecal incontinence, fecal retention, painful or hard bowel movements, or large-diameter feces [1]. FCC accounts for the vast majority of constipation in children and refers to constipation without a clear cause [34]. The pathogenesis of FCC has not yet been elucidated. At present, it is believed that the etiology of FCC is related to colon and rectal dysmotility, pelvic floor dysfunction, psychosocial factors, and abnormal gastrointestinal regulatory peptides. During the development of FCC, with the accumulation of intestinal feces, water is continuously absorbed. Simultaneously, bacteria in the colon, particularly *Enterococcus, Escherichia* coli, and *Klebsiella* [35], overproliferate and ferment with carbohydrates, resulting in increased gas release, which in turn aggravates the symptoms of abdominal distension, bloating, abdominal discomfort, flatulence, diarrhea, and/or constipation. In severe cases, these bacteria may also cause intestinal villi atrophy, malabsorption, and fat-soluble vitamin deficiency [36]. In this process, bacteria and stool stimulate the intestines to increase in volume, which leads to inflammation, and this occurrence of inflammation will continue to increase the occurrence of constipation and induce the formation of a serious “constipation-inflammation-aggravated constipation” promotion model [36, 37]. Our research found that the stimulation of BL25 and ST25 appears to affect the occurrence of inflammation, as mainly reflected by the enrichment of Th17-cell differentiation, the NF-kappa B signaling pathway and the Toll-like receptor signaling pathway in the KEGG clusters and the inflammatory pathway in the local STRING network clusters.

The article "Network-Based Elaboration of the Efficacy of the Dachangshu (BL25) and Tianshu (ST25) Points in the Treatment of Functional Constipation in Children through Inflammation, Adipocytokine, or Leptin Pathways" was retracted in 2023. Reasons: signs of a paper mill; suspected computer-generated content; unreliable results or conclusions; concerns about the data.

As one of the CD4+ T-cell subsets, Th17 cells play a dual role in the pathogenesis of inflammation-related bowel disease (mainly proinflammatory). These cells can not only protect the intestinal mucosa by maintaining the balance of the immune microenvironment but also aggravate the intestinal inflammatory response through proinflammatory cytokines. Th17 cells can secrete IL-17, IL-21, and IL-22 and the proinflammatory cytokines IL-1, IL-6, IL-18, and TNF-*α* [38]. Among these factors, IL-17 is an important cytokine secreted by Th17 cells that can induce inflammation and aggravate tissue damage. The IL-17A subtype of IL-17 can act on a variety of cells (such as epithelial cells and fibroblasts) to secrete chemokines and cytokines. Simultaneously, this subtype can promote the proliferation and maturation of neutrophils, macrophages, and lymphocytes through cell colony-stimulating factors and chemokines [39]. The potential regulatory effect of BL25 and ST25 on Th17-cell differentiation appears to be very important for FCC-induced intestinal inflammation.

In addition, the NF-kappa B signaling pathway has long been regarded as a typical proinflammatory signaling pathway, mainly based on the role of NF-kappa B in the expression of proinflammatory genes, including cytokines, chemokines, and adhesion molecules [21]. Due to the extensive role of the NF-kappa B signaling pathway in cell proliferation, apoptosis, angiogenesis, inflammation, metastasis, and drug resistance [40], the NF-kappa B signaling pathway has also been explored in various diseases, including enteritis [41], ulcerative colitis [42], intestinal flora [43], and rectal cancer [40]. Similar to the NF-kappa B signaling pathway, the Toll-like receptor signaling pathway can also trigger a series of cellular responses and thereby elicits a range of cellular responses, including proliferation, anergy, and apoptosis [44]. The Toll-like receptor signaling pathway can also regulate the enteric nervous system, neurochemical coding, and enteric neuromuscular function to regulate intestinal inflammation [22]. Moreover, the Toll-like receptor signaling pathway can regulate the NF-kappa B signaling pathway and further affect intestinal function [45]. In summary, this study found that BL25 and ST25 exert potential regulatory effects on Th17-cell differentiation, the NF-kappa B signaling pathway and the Toll-like receptor signaling pathway, which further affects the “constipation-inflammation-aggravated constipation” model and thereby reduces the degree of FCC aggravation.

#### 4.2.2. BL25 and ST25 Regulate FCC through Adipocytokine or Leptin

Adipocytokines are peptides that signal the functional status of the adipose tissue to the targets in the brain, liver, pancreas, immune system, vasculature, muscle, and other tissues. Adipokines, including leptin, adiponectin, fibroblast growth factor 21, retinol-binding protein 4, dipeptidyl peptidase 4, bone morphogenetic protein-4, BMP-7, vaspin, apelin, and proanulin, play an important role in the function of the adipose tissue and obesity-related diseases. Leptin is a 16-kDa protein composed of 167 amino acids [46]. Leptin is secreted by adipocytes and plays an important role in regulating satiety, appetite, food intake, reproductive function, fertility, puberty, activity, energy expenditure, atherosclerosis [46, 47], and fetal growth [48] through leptin receptors on target cells. In the hypothalamus, leptin can also reduce the synthesis of orexin, which subsequently leads to a decrease in appetite [46]. In addition, leptin may play a role in insulin sensitization and is considered an important regulator of *β* cells. Due to the ability of recombinant leptin to reduce appetite under normal or low circulating leptin conditions, recombinant leptin has been developed as a weight-loss drug for the treatment of obesity [47, 49].

The article "Network-Based Elaboration of the Efficacy of the Dachangshu (BL25) and Tianshu (ST25) Points in the Treatment of Functional Constipation in Children through Inflammation, Adipocytokine, or Leptin Pathways" was retracted in 2023. Reasons: signs of a paper mill; suspected computer-generated content; unreliable results or conclusions; concerns about the data.

At present, weight loss is considered an alarm symptom of gastrointestinal disease, but the relationship between obesity and gastrointestinal symptoms is unclear [50]. However, a meta-analysis of gastrointestinal symptoms and obesity (analysis of studies from 1950 to November 2011) found a strong correlation between obesity and incomplete evacuation [50]. Another meta-analysis involving 20 studies showed that obesity is associated with fecal incontinence and diarrhea rates [51]. Although the correlation between obesity and constipation cannot be accurately concluded, a close relationship between obesity and gastrointestinal symptoms has been proven. This study found that BL25 and ST25 have the potential to regulate the adipocytokine signaling pathway, orexin receptor family, and prepro-orexin, including signaling by leptin and erythropoietin-mediated activation of phospholipase *C* gamma (PLCG). This finding may indicate that BL25 and ST25 can regulate FCC through adipocytokine or leptin, and although more evidence is needed, this study at least provides a new idea.

#### 4.2.3. BL25 and ST25 Regulate FCC Function and Other Diseases

Approximately less than 5% of children with constipation have organic changes, and these organic changes include anorectal malformations, megacolon, neurological abnormalities, or endocrine and metabolic disorders. More than 95% of children with constipation have no obvious organic causes and are considered to have FCC. However, this study found that leishmaniasis, Chagas disease (American trypanosomiasis), malaria, African trypanosomiasis, toxoplasmosis, hepatitis B, osteoclast differentiation, and measles may be related to FCC, but the relationship between these diseases and FCC is currently poorly understood. However, according to the theory of Chinese medicine, humans should be considered as a whole, and the various tissues and organs of the human body can cooperate with each other to complete various complex physiological functions. Therefore, it does not seem impossible that the occurrence of one disease will eventually cause the occurrence of another disease. Of course, more research is needed on the internal links between these diseases and FCC. We only provide the current results obtained through bioinformatics analysis, and we expect that more scholars will explore and further decipher these findings.

The article "Network-Based Elaboration of the Efficacy of the Dachangshu (BL25) and Tianshu (ST25) Points in the Treatment of Functional Constipation in Children through Inflammation, Adipocytokine, or Leptin Pathways" was retracted in 2023. Reasons: signs of a paper mill; suspected computer-generated content; unreliable results or conclusions; concerns about the data.

Our PPI analysis also revealed that the proteins involved in the abovementioned regulatory functions are NFKBIA, RELA, TNF, IKBKB, IRAK1, TLR4, MYD88, TNFRSF1A, IL1R1, TLR2, IL1B, TRAF6, and TNFRSF1B, as shown in Figure 7.

### 4.3. Innovative Attempts for Using BL25 and ST25 for FCC

Any strong or weak external stimulus can alter the physiological functions of the human body. The most basic changes are those related to protein conformation and output caused by gene expression, which result in various positive or negative bodily states. Based on this information, the stimulation of BL25 and ST25 will inevitably change the human body, and exploring the changes in genes or proteins produced after the stimulation of BL25 and ST25 is thus meaningful.

Based on the existing evidence, this study revealed the targets of BL25 and ST25 and performed enrichment analyses, as shown in Figure 8, and the research thus represents a new attempt to explore the mechanism of acupoints. We hope to provide new ideas and methods for the development of acupuncture strategies.

## 5. Conclusion

At present, there are many difficulties in acupuncture research, such as the difficulty of determining the targets of acupoints, and the theory of acupoint compatibility has not been effectively proven. This research explored published articles, collected the existing BL25 and ST25 targets for further research, and explored the connotation of combinations of back-shu and front-mu points for TCM. This research draws the following conclusions:

1. BL25 and ST25 exert a synergistic effect.
2. The pathway through which BL25 and ST25 regulate FCC is closely related to inflammation and adipocytokine or leptin.
3. The findings indirectly prove the usability of the method of matching points based on the back-shu and front-mu point combination.

In short, this study provides a new method and idea for exploring the mechanism induced by acupuncture points and provides a new research direction for the modernization of Chinese medicine, particularly acupuncture and moxibustion.

## Figures and Tables

**Figure 1:** Workflow for the regulation of FCC by BL25 and ST25.

**Figure 2:** BL25 and ST25 target information. The BL25 targets are shown in light purple, the ST25 targets are shown in wine red, and the common BL25 and ST25 targets are shown in lime green.

**Figure 3:** Venn diagram of FCC genes and acupoint targets.

**Figure 4:** Top 20 terms identified from the KEGG enrichment analysis.

**Figure 5:** Top 20 items identified by local STRING network cluster enrichment analysis.

The article "Network-Based Elaboration of the Efficacy of the Dachangshu (BL25) and Tianshu (ST25) Points in the Treatment of Functional Constipation in Children through Inflammation, Adipocytokine, or Leptin Pathways" was retracted in 2023. Reasons: signs of a paper mill; suspected computer-generated content; unreliable results or conclusions; concerns about the data.

**Figure 6:** Pathway-target relationship network.

**Figure 7:** Mechanism of action of BL25 and ST25. The red color indicates the pathways, and the blue color indicates the targets.

**Figure 8:** Roadmap for this research.

## Data Availability

The data used to support the findings of this study are included within the supplementary information files.

## Supplementary Materials

Supplementary Materials Supplementary file 1: acupoints and disease-related targets. Supplementary file 2: KEGG enrichment analysis of 141 items. Supplementary file 3: local STRING network cluster enrichment analysis of 59 items.
